The article "Childhood nosocomial viral acute respiratory tract infections in teaching hospital Anuradhapura, Sri Lanka" was retracted in 2021. Reasons: unreliable data; lack of ethics approval or compliance.

# Childhood nosocomial viral acute respiratory tract infections in teaching hospital Anuradhapura, Sri Lanka

**DOI:** 10.1186/s13104-019-4624-2

**Published:** 2019-09-14

**Authors:** Jayaweera Arachchige Asela Sampath Jayaweera, Mohammed Reyes

**Affiliations:** 1 Department of Microbiology, Faculty of Medicine and Allied Sciences, Rajarata University of Sri Lanka, Saliyapura, 50008 Sri Lanka; 2 Department of Pediatrics, Faculty of Medicine and Allied Sciences, Rajarata University of Sri Lanka, Saliyapura, 50008 Sri Lanka

**Keywords:** Childhood, Nosocomial: viral acute respiratory tract infections, Respiratory syncytial virus and risk factors

## Abstract

**Objectives:**

We have assessed the risk factors for the occurrence of hospital-acquired (HA) and community-acquired (CA) viral acute respiratory tract infections (ARTIs) in children. Children (1–60 months) who were having ARTI on admission (CA) and develops ARTI following 48 h after admission or 3 days of discharge (HA) were included. Indirect immunofluorescence assay (IFA) was performed and multivariable analyses were done to determine the risk factors for the development of viral CA and HA-ARTI.

**Results:**

Total of 818 with ARTIs, 226 (27.6%) RSV cases were detected. Out of 226, 86 (38.0%) HA-RSV cases were detected. CA-viral-ARTI was significantly high (p < 0.05). Compared to CA-RSV-ARTI immunodeficiency, seizures, trisomy-21 and congenital heart disease (CHD) were having 2.3, 3.2, 1.8- and 2.2-times risk for acquiring HA-RSV respectively. The number of deaths was significantly high following HA-RSV. The associated burden was significant following HA-RSV and it was 429.77 disability-adjusted life years. Children who are having immunodeficiency, CHD, seizure episodes and trisomy 21 would lead to the acquisition of nosocomial RSV infections in great. Adherence to meticulous infection control practices will be helpful to minimize the HA-viral ARTIs in great.

## Introduction

Hospital-acquired infections (HAI) are associated with a great deal of morbidity and mortality [1, 2]. HAIs affect 10% of patients admitted to the hospital and are more prevalent in the intensive care facility [3, 4]. Also, it is common inward set up as well [5].

Hospital-acquired infections are most commonly associated with indwelling medical devices and surgical procedures. Out of HAIs pneumonia and bloodstream infections are the most lethal while urinary tract infections are the most common [6, 7]. Only a few studies on viral nosocomial acute respiratory tract infections (ARTI) were described. The first published description of nosocomial ARTI was in 1937. It was following the respiratory syncytial virus (RSV) [8]. In children viral ARTI is common and its associated burden is high [9].

The article "Childhood nosocomial viral acute respiratory tract infections in teaching hospital Anuradhapura, Sri Lanka" was retracted in 2021. Reasons: unreliable data; lack of ethics approval or compliance.

For instance, while getting care for other diseases many patients probably acquired respiratory infections [10]. Therefore, is troublesome to spot the prevalence of any of nosocomial viral infection. Great awareness and adherence to meticulous infection control practices are the mainstays of reducing HAIs. In this study, we have assessed the risk factors for the occurrence of nosocomial and community-acquired viral ARTIs in children 1 month to 5 years of age.

## Main text

### Study design

This was a cross-sectional study.

### Study site

The study was performed at the children’s ward of the Professorial Unit, Teaching Hospital Anuradhapura, (THA), Sri Lanka from March 2015 to August 2016.

### Study population

Children aged from 1 to 60 months and who having ARTI (community-acquired as the control group) on admission were included. Further, (child aged 1–60 months) who has admitted for different diseases and develops ARTI following 48 h after admission or 3 days of discharge (HAI) were also included (as test group). For the recruitment of the latter group, pieces of advice were given and a telephone interview was conducted on days-2 and 3 following discharge by the investigator to assess the development of ARTI within 3 days. ARTI cases include all children were having severe acute respiratory tract infection (SARI) on admission and development of ARTI following discharge [5]. An investigator administered questionnaire was used to collect demography and clinical data.

All subjects that fulfill inclusion criteria nasopharyngeal aspirate (NPAs) were collected with the help of recommended mucus extractor by the investigators. Indirect immunofluorescence assay (IFA) [specificity was 99% and sensitivity was 38%] was performed by DAKO IMAGEN™ (United Kingdom), respiratory screening reagents for eight respiratory viruses and viral typing was done for each of respiratory syncytial virus (RSV), adeno (AV), parainfluenza 1, 2 and 3 (PIV 1, 2 and 3), influenza A (Inf A) and B (Inf B) and Human metapneumovirus (hMPV) viruses using monoclonal antibodies DAKO IMAGEN™ (United Kingdom) [11].

### Statistical analysis

The risk factor analysis was performed using the Chi-squared test and stepwise logistic regression. Following univariate analysis, the variables having a p-value of < 0.05 were included in multivariate analysis. The factors having odds ratios with 95% confident interval (CI)s that did not include 1.0 were regarded as significant. Gender, ethnicity, weight (kg), hemoglobin %, chronic malnutrition (height-for-age ≤ 2SD was taken while weight-for-age ≤ 2SD to assess the status of malnutrition), pre-maturity, low birth weight (< 1500 g), mode of delivery (normal vaginal or lower segment cesarean section) and having medical conditions (congenital heart disease-CHD; chronic lung disease-CLD, asthma, cystic fibrosis), development of seizure in at ward among known epilepticus and genetic disorders; Down’s syndrome-trisomy 21; neuromuscular disorders and pre-existing respiratory tract morbidity, passive smoking (the involuntary inhaling of smoke from other people’s cigarettes, cigars, or pipes produced by child’s father or any other relation/s at the vicinity of child—here we have taken indoor smoking), having house hold pets, presence of indoor (fire woods used for cooking and houses do not have chimney) and outdoor air pollution (following construction activities having outdoor dusty nature where child plays or lives), crowding (child’s living area < 24 m^2^ and > 2 personal living in the area) [12, 13] guardian’s/parent’s education (< grade 8, up to advanced level and graduates), experience as a caregiver (first child or experience in caring > 1 child) and occupation. The statistical software SAS Version 9.1 was used [14].

The article "Childhood nosocomial viral acute respiratory tract infections in teaching hospital Anuradhapura, Sri Lanka" was retracted in 2021. Reasons: unreliable data; lack of ethics approval or compliance.

## Results

### Nosocomial viral ARTIs

A total of 818 children with ARTIs, 320 (39.5%) positive samples were detected by using IFA. Out of 320 viral ARTIs, 226 (70.6%) were positive for RSV. From that 86 (38.0%) nosocomial RSV was detected. Period prevalence of nosocomial and community-acquired RSV, PIV-1, PIV-2 and PIV-3, AV, Inf-A, Inf-B and hMPV in children with ARTI was displayed in Table 1. Compared to other viruses, nosocomial RSV was significantly common (p = 0.001). Recurrent inward admissions following ARTI in was 37 out of 818 (4.5%) cases. From that RSV was (13.8%) detected in 29 cases (3.5%). RSV was significantly associated with recurrence ARTI admissions (p = 0.04).

**Table 1:** Incidence/100,000-person years for hospital acquired and community acquired RSV, PIV-1, PIV-2 and PIV-3, AV, Inf-A, Inf-B and hMPV among of children with ARTI compared to overall incidence

Age group (months)	Viral aetiologies								*p* value and comments
	RSV	PIV-1	PIV-2	PIV-3	AV	Inf-A	Inf-B	hMPV	
Nosocomial	8.41	0.18	0.44	0.10	0.67	0.54	0.03	0.30	Compared to other viruses, nosocomial RSV was significantly common (p = 0.001); All of community acquired viral ARTI was significantly higher than nosocomial viral infections
CA	22.82	1.21	2.01	1.20	2.13	1.01	1.03	1.01	
Period prevalence over 1 year	31.33	1.39	2.45	1.30	2.80	1.55	1.06	1.31	

Community acquired (CA), respiratory syncytial virus (RSV), adeno (AV), parainfluenza 1, 2 and 3 (PIV 1, 2 and 3), influenza A (Inf A) and B (Inf B) and human metapneumovirus (hMPV)

p < 0.05 was taken as significant

The article "Childhood nosocomial viral acute respiratory tract infections in teaching hospital Anuradhapura, Sri Lanka" was retracted in 2021. Reasons: unreliable data; lack of ethics approval or compliance.

### Risk factors for the development of HA and CA-RSV

Since RSV was predominant viral etiology, RSV was included in risk factor analysis. Most of the assessed risk factors for the acquisition of both hospital and community-acquired RSV were similar and not statistically significant (p > 0.05). Child delivered following lower segmental caesarian section having 2 times risk in acquisition of HA-RSV in the first 2 years of life compared to CA-RSV ARTI. Outdoor air pollution is having 3.2 times the risk for acquiring CA-RSV infection compared to HA-RSV ARTI.

Having any type of known immunodeficiency, development of seizures, a child with trisomy-21 and CHD was having 2.3, 3.2, 1.8- and 2,2-times significant risk for acquiring HA-RSV infection compared to CA-RSV ARTI respectively. Further, having a urinary tract infection 3.1; having central nervous tract infection 2.2 and having gastro-enteritis poses 1.8 times the risk for acquiring HA-RSV infection (Table 2).

**Table 2:** Risk factors assessment for acquisition of community acquired (CA) and hospital acquired (HA)-RSV

	CA-RSV (140)	HA-RSV (86)
Number of pt. with co infections^a^	9	4
Risk factors		
Malnutrition (weight-for-age *z*-score > − 2)	–	–
Male sex	–	–
Low birth weight (< 2500 g)	–	–
Mode of delivery—LSCS	–	2.0 (0.04)
Outdoor air pollution	3.2 (0.04)	–
Indoor air pollution	–	–
Passive smoking	–	–
Non-exclusive breastfeeding (during the first 4 months of life)	–	–
Lack of measles immunization (within the first 12 months of life)	–	–
Crowding	–	–
Concomitant diseases		
Urinary tract infection	–	3.1 (0.03)
Infection in central nervous system	–	2.2 (0.04)
Gastro-enteritis	–	1.8 (0.03)
Congenital heart diseases	–	2.2 (0.04)
Asthma	–	–
Immunodeficiency^b^	–	2.3 (0.04)
Development of seizure in at ward in known epileptics	–	3.2 (0.04)
Mother’s experience as a caregiver	–	–
Mother’s education	–	–
Day-care attendance	–	–
Relative humidity (%)	–	–
Rain days/month	–	–
Trisomy 21	–	1.8 (0.03)
Birth order > 3	–	–

^a^RSV co-infection with other viruses were not included in risk factor analysis

^b^Subjects were considered immunocompromised if they had any of the following: positive HIV test, report of HIV infection; receiving a prolonged course of steroids or other immunomodulatory medications; neutropenia during the hospitalization; or undergoing active chemotherapy during the hospitalization. Significant odds ratio with p value was given

### Associated burden following viral ARTIs

The case-fatality ratio for HA-RSV infection was 16.7% while following CA-RSV it was 2.27% (p = 0.01). Furthermore, all mortalities were associated with RSV associated pneumonia. The number of deaths was high following HA-RSV. Further, the associated burden was significant following HA-RSV and it was 429.77 and 242.06 DALYs following HA and CA-RSV respectively. Using multiple logistic regression analysis (Table 3). Down’s syndrome (trisomy 21) (OR 4.20, 95% CI 1.23–11.76; *p* = 0.03), congenital cardiac diseases (OR 3.46, 95% CI 1.29–10.27; *p* = 0.01), having urinary tract infections (OR 5.46, 95% CI 1.89–22.27; *p* = 0.001) and intensive care were (OR 3.46, 95% CI 1.79–11.27; *p* = 0.01) predictive factors for death following HA-RSV. Further, delivery following the lower segment caesarian section (OR 2.16, 95% CI 1.19–4.12; *p* = 0.03) was a predictive factor for death following CA-RSV.

The article "Childhood nosocomial viral acute respiratory tract infections in teaching hospital Anuradhapura, Sri Lanka" was retracted in 2021. Reasons: unreliable data; lack of ethics approval or compliance.

**Table 3:** Mortality and morbidity in children with HA RSV associated ARTIs

Parameters	HA-RSV	CA-RSV	p value and comment
Total number of children with ARTI	86	140	0.001
Number of deaths	8	3	0.01
Associated risk			
Infectious			
UTI	4	0	0.001
Non-infectious			
CHD	2	0	0.01
Trisomy 21	2	0	0.01
Mode of delivery—LSCS	0	2	0.03
ICU care	6	1	0.01
DALYs	429.77	242.06	0.01

*DALYs* disability adjusted life years

p < 0.05 was taken as significant

## Discussion

Respiratory viruses are important pathogens causing hospital-acquired infections [15, 16]. Several hypothetical explanations were specifically described as the nosocomial extinction of RSV in previous studies. For decades, it has been known that viral nosocomial ARTIs is a particular problem in pediatric patients [17]. In our study, RSV was predominantly (87.5%) associated with nosocomial ARTIs. Detailed studies of non-influenza nosocomial respiratory viral infections are limited. A recent study conducted at nonepidemic settings in the United States found that the rhinovirus and/or enterovirus were the predominant nosocomial viruses in children and adults with ARTIs [18]. A previous prospective cohort study demonstrated that rhinovirus was the most commonly detected virus among children with viral respiratory infections, and approximately 20% of these infections were hospital-acquired [19]. Impact, 73% of nosocomial respiratory infections among children were due to rhinovirus [20]. In here, we haven’t tested rhino and enteroviruses. So, we may have missed a fair amount of nosocomial viral ARTIs. However, another study conducted in children under 5 years of age found that RSV and influenza were associated with 51% and 19% of such cases, respectively [21].

Once considered the risk factors; modifiable risk factors, outdoor air pollution and mode of delivery (following caesarian section) were significantly contributed to the acquisition of HA-RSV [22]. Outdoor dusty nature was predominant in the study period where most of the rural and urban road construction and development were undertaken. Delivery following the caesarian section would lead to a low level of immunity and adaptability thus warrant a higher tendency for the development of infections [23]. Passive smoking and indoor air pollution neither risk or protective factors for the acquisition of HA or CA-RSV. Perhaps these could be risk factors for the occurrence of any viral ARTIs.

The article "Childhood nosocomial viral acute respiratory tract infections in teaching hospital Anuradhapura, Sri Lanka" was retracted in 2021. Reasons: unreliable data; lack of ethics approval or compliance.

More often children get urinary, gastrointestinal tract infections and less frequently get infections in the central nervous system. All conditions could lead to under-nutrition and ended in a low level of immunity thus making vulnerable to respiratory tract infections. Once these children admitted to the health care facility, they are more prone to develop HAI. Children who are having CHD, immunodeficiency, seizure episodes and trisomy 21 would lead to the acquisition of HA-RSV infections in great.

Our study specifically describes the vulnerability of nosocomial RSV infections. Several factors have been discussed about RSV’s high capability of becoming one of the major viral HAI. Outbreaks of RSV infection occur every year and the spread is considerable in the globe. It affects all ages, including healthy and people with underlying conditions. Most bacterial agents causing nosocomial illness, are mostly observed primarily in patients with chronic compromising conditions. The RSV shedding in the respiratory secretions of young children tends to be for longer periods with high titer and in adults shed appreciable quantities of virus for 3 to ≥ 7 days [22, 24]. Finally, RSV in secretions may remain infectious in the environment for periods long enough for transmission on hands and fomites.

Here, children who died from HA-RSV disease had chronic diseases (Down’s syndrome and CHD). Patients with Down’s syndrome are at a greater risk of acquiring RSV-ARTI. Children with Down’s syndrome have an increased rate of comorbidities with both CHD and pulmonary hypertension, which are two independent risk factors for RSV ARTI [25–27]. Further, ICU stay is an independent risk factor for RSV-ARTI. Initially presented to inward care for UTI and later admitted to ICU for further care.

Once compared to nosocomial methicillin resistance *Staphylococcus aureus* and candidiasis, the risk of mortality is less in HA-RSV [28, 29]. Contrary the morbidity is high because the incidence is high and associated burden to the family, the society finally to the country is high. This is mainly because it is prevalent among children so the guardian has to stay with the child and provision of care is demanding [24, 25].

Respiratory syncytial virus is mainly spread following close contact with aerosols of infectious respiratory secretions and medical staff is at risk of acquiring as well as spreading the virus. RSV is a labile virus and is promptly inactivated following contact with alcohol, detergents, and antibacterial soaps [13, 21]. Thus hand-washing probably plays the most important part in infection control. Although there are various barrier methods, the isolation of RSV-positive patients in single rooms or cohorting is recommended [30]. Central to such practice is to make healthcare personnel as well as parents/guardians of patients aware of characteristics, transmission, and risk factors for the occurrence of nosocomial RSV-ARTIs.

The article "Childhood nosocomial viral acute respiratory tract infections in teaching hospital Anuradhapura, Sri Lanka" was retracted in 2021. Reasons: unreliable data; lack of ethics approval or compliance.

## Limitations

It is unclear whether all of the viruses identified were the cause of active infection, or whether their presence in some cases reflected respiratory tract colonization or recent respiratory viral infection. Further, in Sri Lanka, Ribavirin and Palivizumab therapy are not offered and only supportive care with the prevention of secondary bacterial pneumonia by empiric broad-spectrum antibiotics was prescribed for RSV infections [26]. Based on this viral etiological diagnosis doesn’t add therapeutic value to the patient. We haven’t performed molecular diagnostics for virus detection would reduce the number of exact HA-viral ARTIs. We haven’t assessed the infection control practices and the occurrence of HA-RSV ARTI.

## Data Availability

The datasets used and/or analyzed during the current study are available from the corresponding author on reasonable request.

## Abbreviations

HA: hospital-acquired
CA: community-acquired
ARTI: viral acute respiratory tract infections
IFA: indirect immunofluorescence assay
HAI: hospital-acquired infections
NPA: nasopharyngeal aspirate
RSV: respiratory syncytial virus
